# Is the Network of World Economic Forum Young Global Leaders Associated With COVID-19 Non-Pharmaceutical Intervention Severity?

**DOI:** 10.7759/cureus.29990

**Published:** 2022-10-06

**Authors:** Rainer J Klement, Harald Walach

**Affiliations:** 1 Department of Radiation Oncology, Leopoldina Hospital Schweinfurt, Schweinfurt, DEU; 2 Research and Development, Change Health Science Institute, Berlin, DEU; 3 Next Society Institute, Kazimieras Simonavicius University, Vilnius, LTU

**Keywords:** health policy and economics, sars-cov-2, covid-19 crisis, non-pharmaceutical interventions, world economic forum

## Abstract

Background

TheWorld Economic Forum (WEF) has spawned a global network of elites called Young Global Leaders (YGLs) with significant influence on large corporations, politics, academia, and media. This article scrutinizes the idea that through this network, the WEF had a significant influence on the scale and scope of the non-pharmaceutical interventions (NPIs) implemented in response to the COVID-19 crisis. We tested for associations between the country-level distribution of YGLs and the intensity and duration of the implemented NPIs summarized by the Government Response Severity Index (GRSI).

Materials and methods

The number and category of YGLs per country was extracted from the WEF website. We also extracted the maximum and median GRSI values for three time periods: (i) the beginning of the first wave of the pandemic (March 1, 2020, to April 30, 2020), (ii) the height of the second wave in Europe (December 1, 2020, to January 31, 2021), and (iii) the approximate first year (March 1, 2020, to January 31, 2021). Being a precondition for causality, any association between the total or category-specific number of YGLs and the GRSI values in each time period was evaluated using Spearman’s ρ correlation coefficients and polynomial regression, respectively.

Results

There was a highly significant positive correlation between the total number of YGLs in a country and the median (ρ = 0.36, p = 2.5×10^-7^) and maximum (ρ = 0.34, p = 1.6×10^-6^) GRSI during the second wave of the pandemic, but not during the first wave. The total number of YGLs was also a significant predictor of higher median GRSI during the second wave of the pandemic in the best-fitting (four-degree) polynomial regression model (p<0.01); additional significant and positive predictor in this model was a country’s location within Europe or South America, respectively (p<0.01). Investigating an influence-weighted number of YGLs in business, politics, and civic society separately yielded no significant associations with NPI severity for any of the three time periods.

Conclusions

As there were significant correlations during the second, but not the first wave of the pandemic, we conclude that the WEF might not have been the origin of but rather an echo-chamber or amplifier for certain opinions and strategies that were formed and implemented during or before the first months of the COVID-19 crisis. Future qualitative studies may reveal putative causal mechanisms underlying our observed correlations.

## Introduction

The declaration of the COVID-19 pandemic by the World Health Organization (WHO) on March 11, 2020 [1], was a cataclysmic event. The more visible problem is the death of countless people that has been associated with SARS-CoV-2 infection, the causative agent of COVID-19. A second, perhaps even more important, part was the response to the pandemic by governments, starting with closures of borders, mask mandates, stay-at-home orders, and business closures and ending with strict curfews. A case can be made that a lot of the secondary problems stem from these political responses, usually called non-pharmaceutical interventions (NPIs) [2,3]. Business closures have affected small businesses that often went out of business, if countries had no relief program in place. Lockdowns and stay-at-home orders have affected poor people more than affluent ones, as in some countries going out for work or buying food is important for sustenance and livelihoods [2]. Although the general idea behind government-mandated NPIs was to “flatten the curve,” and hence to avoid COVID-19 deaths, the collateral damage associated with them might tragically have caused hundreds of thousands secondary deaths [4]. In addition, NPIs were not associated with a reduction of COVID-19 related deaths in several modelling studies [5-7], although Hale et al. found a significant global association between the stringency of NPIs and deaths measured after 28 days [8].

This very mixed picture has given rise to various ideas and theories as to why governments stuck to NPIs, although many of these have been found to be ineffective or irrelevant quite early on. Some people find sinister motives behind this situation and have come up with the idea that rich elites have attempted a silent takeover of countries and democracies to foster the benefit of big corporations [9]. The World Economic Forum (WEF) is often mentioned as one of the putative forces. The WEF can be conceptualized as a think tank situated in-between the fields of business, politics, academia, and media, and it has also been identified as a transnational space for the formation of a global capitalist or technocratic elite [10-12]. The WEF may hence be counted among the “transnational policy networks” that exert “disproportionate influence over policy design and implementation on issues of global importance” [13]. This is exemplified by an 2017 interview with its founder, Professor Klaus Schwab, who correspondingly said: "What we are very proud of, is that we penetrate the global cabinets of countries with our World Economic Forum Young Global Leaders" [14]. Schwab also published a COVID-19-related book entitled “The Great Reset” in 2020 [15]. On first sight, this book could be seen as a description of potential opportunities rather than a sinister plan, in line with the general tendency of the WEF to have a positive outlook and to benefit the world, to “make the world a better place”, improving living and working conditions by marrying economic growth with ecologic and social sustainability [12,16,17]. Yet, an in-depth analysis shows that in its essence the “Great Reset” also contains normative ideas, the implementation of which would transform our liberal democracies into top-down managed societies with the new normative primacy of “health” as the absolute value, conceived for individuals, economy, politics, and the planet [18]. In addition, Schwab could have anticipated the COVID-19 pandemic because together with the Bill & Melinda Gates Foundation, the WEF hosted a major pandemic simulation exercise called “Event 201” on October 18, 2019, just a few months before the start of the COVID-19 pandemic [19].

According to some authors [20], it is difficult to test and challenge a “conspiracy theory” of the kind that the WEF is one of the causative players if not in the pandemic itself then in the rolling out of NPIs worldwide; however, deHaven-Smith pointed out that “political conspiracies in high office do, in fact, happen” ([21], p. 6), so it should be possibly to objectively define and test the above theory about the WEF. We attempt here to approach the question empirically. Even though the WEF might be an important hub in the global discursive landscape, an active role in promoting NPIs might stem from a well-meaning intent because a majority and some important opinion leaders in the scientific community believe in the effectiveness of NPIs [22].

Our study starts from the assumption that if the WEF does play a role, it would do so by its generic and unique placement as a worldwide network of high-profile organizations and their representatives. There are various channels of influence. One is through the 1,000 biggest corporations that are members of the WEF and fund it [16]. Another is through the approximately 1,250 Young Global Leaders (YGLs) who, since 2016, have undergone the YGL training and are thus assumed to act as ambassadors of the WEF values and ideas. These YGLs are distributed across countries and have various roles, from administrative-political to economic and public service ones. For instance, in Germany, former chancellor Angela Merkel, former secretary of health Jens Spahn, and current foreign secretary Annalena Baerbock have undergone the WEF YGL training [23], as has France’s president Macron. If the WEF plays a role at all, then there should be an association between the influence level of YGLs and/or their number in a country and the NPI response. Hence, in this study, we address the research question: *Is the number and the gravitas of YGLs in a country associated with the country’s NPI in the first phases of the pandemic in 2020*? We deliberately focus on the first phases of the pandemic, as later stages might comprise a mix of motives.

## Materials and methods

Research design

The protocol of this study with definition of data and description of analytical procedures was developed and posted in advance at the Open Science Foundation platform (https://osf.io/reqn3/). Briefly, this was a quantitative analysis testing a set of pre-specified hypotheses by assuming that a causal influence of YGLs on shaping policy responses to the COVID-19 pandemic, if indeed present, may yield a correlation between the number or another metric of YGLs and the severity of NPIs.

A preprint containing the results of this analysis was posted on the Social Science Research Network platform on September 12, 2022 [24].

Data

We extracted the number and types of YGLs per country from the WEF’s website; we used the year 2016 as a cutoff date because we assumed that a more recent training would mean a more intimate involvement with the WEF. For defining a YGL type, we made a generic categorization into the following eight categories: (i) academia, (ii) arts and media, (iii) business (corporations), (iv) civic society (non-governmental organizations [NGOs], advocacy groups, and similar civic organizations), (v) political party members, (vi) politics (administration, government, parliaments, and public offices), (vii) religion, and (viii) sports. We used the categorization presented on the WEF page itself. Where it was obviously wrong, we corrected it.

We also introduced a quality rating to judge the YGL’s putative influence. To this aim, a weight of 0.33 was assigned to YGLs with a generic influence (member of a corporation, political arena), 0.66 to those with a stronger influence (secretary of state, member of the board), and 1 to YGLs having supreme influence (presidents of state or business leaders).

The Government Response Severity Index (GRSI) and the population size of each country were retrieved from a spreadsheet downloaded from the Our World in Data (OWID) website (https://ourworldindata.org/covid-vaccinations, accessed on April 12, 2022). We extracted the maximum and median strength of NPIs during the beginning of the first wave of the pandemic (March 1, 2020, to April 30, 2020), the height of the second wave in Europe (December 1, 2020, to January 31, 2021) [25], as well as for the total time span from March 1, 2020, to January 31, 2021. For countries for which GRSIs were available but no YGL could be found, the number and gravitas of YGLs for this country was set to zero. The criterion for including countries into this analysis was the availability of at least one Oxford GRSI within the timeframe from March 2020 to January 2021. The GRSI is updated daily and measures the strength of a country’s NPIs on a scale from 0 to 100 [26].

The population number of all countries included in the analysis was used to calculate population-standardized numbers of YGLs for sensitivity analysis.

Analytical procedures and hypotheses

If YGLs would have a causal influence on the severity of NPIs in a given country, an association of the number of YGLs or their strength of influence with the GRSI would be expected as a precondition for causality. Hence, we posed a few straightforward hypotheses to test for such associations.

The most generic hypothesis (H1) was that the WEF functions as a large amplifier network for “his master’s voice” [12], whoever the master is supposed to be (see Phillips [27] and Röper [28] for evidence that the master is a network of a small number of global power elites, financial companies, and NGOs). This was tested by a simple correlation between the number of YGLs in a country and the maximum and median strength of NPIs within each of the three timeframes considered. Without making assumptions about the probability distribution of median and maximum GRSIs, we used non-parametric Spearman’s rank correlation coefficients (ρ) to measure the strength of association.

The second, more specific hypothesis (H2) was that the more influential YGLs are, the stronger the NPIs in a country, if they have any influence at all. This was tested by using the weighted number of YGLs per country as defined above, i.e., each YGL was counted as 0.33, 0.66, or 1 depending on the putative strength of his/her influence. The same correlation analysis that we used to test hypothesis H1 was then performed, but using the weighted instead of total number of YGLs per country.

A third, more specific hypothesis (H3) considered the case that business interests and political interests may be divergent. In this case, one would expect that the influence of business leaders and that of political and civic society leaders is different. This hypothesis was tested by a linear regression approach, in which the weighted number of YGLs belonging to the categories of politics, economy, and civic society were used together to predict the maximum and the median strength of NPIs per country. We accounted for the possibility that different COVID-19 phases had different impacts in different continents by including continent as a categorical variable having five possible values (Africa as a reference, Asia, Europe, North America, Oceania, and South America).

All analyses were considered as supporting or refuting plausibility assumptions about the hypothesized associations. Since the hypotheses assumed positive correlations, the null hypothesis for purely correlational analyses was that of a negative or no association (Spearman’s ρ≤0). A positive correlation was defined as Spearman’s ρ>0.3 with an associated p-value of ≤0.005 [29]. For regression analysis, statistical significance of a predictor was defined as p<0.01, and models were compared by the bias-corrected Akaike Information Criterion (AICc) [30]. All analyses were performed in R version 4.0.2.

## Results

Characteristics of included countries

The OWID database yielded GRSI data for 182 countries. Information about the strength of NPIs was available for all of these countries during the second wave of the pandemic (December 2020 to January 2021), but was unknown in four countries for the first wave (March to April 2020). Of these 182 countries, 109 hosted at least one YGL according to the WEF webpage information.

Table 1 provides information on the number and type of YGLs per country, the median and maximum GRSI values, and population sizes. It is evident that the severity of NPIs was significantly greater during the first wave compared to the second wave of the pandemic which was confirmed by a paired Wilcoxon rank sum test yielding p<2.2×10^-16^. The spectrum of YGL types was dominated by individuals in businesses such as companies or corporations, followed by academia and civic society. On average, there were almost seven YGLs per country, although more than half of the countries had none (N=73) or only one (N=25) YGL.

**Table 1:** Baseline characteristics of the 182 countries included in the analysis GRSI, Government Response Severity Index; YGL, Young Global Leader

Variable	Median (range)	Mean (standard deviation)
Total number of YGLs	1 (0-313)	6.8 (25.6)
Weighted number of YGLs	0.75 (0-179)	4.0 (14.6)
YGL type		
Academia	0 (0-32)	0.5 (2.5)
Arts and media	0 (0-11)	0.3 (1.3)
Business	2 (0-247)	5.7 (19.7)
Civic society	1 (0-14)	0.9 (1.7)
Political party	0 (0-1)	0.03 (0.18)
Politics	2 (0-8)	1.4 (1.3)
Religion	0 (0-1)	0.01 (0.10)
Sports	0 (0-1)	0.005 (0.07)
Median GRSI		
March 1, 2020, to April 30, 2020	80.09 (8.33-100)	77.02 (16.25)
December 1, 2020, to January 31, 2021	58.56 (6.48-89.81)	56.16 (18.30)
March 1, 2020, to January 31, 2021	61.57 (13.89-89.81)	59.94 (16.43)
Maximum GRSI		
March 1, 2020, to April 30, 2020	85.42 (13.89-100)	82.33 (14.19)
December 1, 2020, to January 31, 2021	65.28 (8.33-90.74)	61.81 (18.54)
March 1, 2020, to January 31, 2021	87.04 (18.06-100)	83.32 (14.46)
Population size	1.0×10^7^ (3.4×10^4^ – 1.4×10^9^)	4.3×10^7^ (1.5×10^8^)
Continent		
Africa	50	
Asia	46	
Europe	44	
North America	23	
Oceania	7	
South America	12	

Associations between YGLs and NPIs

The results of testing hypothesis H1 are shown in Table 2. There was a highly significant positive correlation between the number of YGLs in a country and the median and maximum GRSI during the second wave of the pandemic, but not during the first wave. Concerning the whole timeframe from March 2020 until January 2021, the correlation between the number of YGLs and median GRIS was also significant, but not very strong (ρ=0.26). Very similar results were obtained when testing hypothesis H2, which considered the putative influence of YGLs by using a weighted number per country (Table 3). In contrast, when using the total number of YGLs standardized to 100,000 inhabitants of a country, the association became somewhat weaker (Table 4). Because the correlations were negligible during the first wave, but highly significant during the second wave, we investigated how the correlation coefficients changed during the first year of the pandemic. As shown in Figure 1, the correlation became significant not until September/October 2020, and its numerical value reached >0.3 during the following months.

**Table 2:** Spearman’s rank correlation coefficients for testing hypothesis H1 P-values are one-sided with the null hypothesis tested displaying a negative or no association and the alternative hypothesis displaying a positive association (ρ>0). * p<0.005 (statistically significant). GRSI, Government Response Severity Index

Period	Median GRSI		Maximum GRSI	
	Spearman’s ρ	p-value	Spearman’s ρ	p-value
March 1, 2020, to April 30, 2020	0.045	0.274	0.031	0.337
December 1, 2020, to January 31, 2021	0.362	2.5×10^-7^*	0.335	1.9×10^-6^*
March 1, 2020, to January 31, 2021	0.257	0.00023*	0.043	0.283

**Table 3:** Spearman’s rank correlation coefficients for testing hypothesis H2 P-values are one-sided with the null hypothesis tested displaying a negative or no association and the alternative hypothesis showing a positive association (ρ>0). *p<0.005 (statistically significant). GRSI, Government Response Severity Index

Period	Median GRSI		Maximum GRSI	
	Spearman’s ρ	p-value	Spearman’s ρ	p-value
March 1, 2020, to April 30, 2020	0.036	0.317	0.030	0.343
December 1, 2020, to January 31, 2021	0.362	2.5×10^-7^*	0.338	1.6×10^-6^*
March 1, 2020, to January 31, 2021	0.256	0.00025*	0.045	0.275

**Table 4:** Spearman’s rank correlation coefficients for testing hypothesis H2 with the number of YGLs standardized to a population of 100,000 P-values are one-sided with the null hypothesis tested being a negative or no association and the alternative hypothesis being a positive association (ρ>0). *p<0.005 (statistically significant). GRSI, Government Response Severity Index

Period	Median GRSI		Maximum GRSI	
	Spearman’s ρ	p-value	Spearman’s ρ	p-value
March 1, 2020, to April 30, 2020	0.045	0.271	0.019	0.401
December 1, 2020, to January 31, 2021	0.314	8.1×10^-6^*	0.291	3.4×10^-5^*
March 1, 2020, to January 31, 2021	0.198	0.0037*	0.039	0.299

**Figure 1:** Change in the strength of correlation between the total number of YGLs in a country and the median GRSI in six 2-month intervals during the first year of the pandemic. GRSI, Government Response Severity Index; YGLs, Young Global Leaders

Finally, we evaluated regression models for their ability to predict the severity of NPIs. Table 5 shows the results for the regression models that were used to test hypothesis H3. The three specific YGL types investigated had no significant impact on the median GRSI in any time period. Among the three types, the weighted number of YGLs in civic society had the largest impact as judged by the size of its regression coefficient, but uncertainties in this estimate were large. During the first wave of the pandemic, continent appeared to play no role as a predictor; in fact, a model fitted without the continent variable was favored by an AICc value, which was 6.25 smaller than the model displayed in Table 5. In contrast, the continental location of a country appeared to play a large role during the second wave of the pandemic, with Europe predicting much more severe restrictions than Africa, followed by South America and Asia. Considering the overall timeframe from March 2020 until January 2021, only South America emerged as a highly significant predictor of a larger median GRSI.

**Table 5:** Regression models for predicting the median GRSI in three time periods according to hypothesis H3 Note that for the period March 1, 2020, to April 30, 2020, four countries were lacking GRSI values. *p<0.01 (statistically significant). AICc, bias-corrected Akaike Information Criterion; GRSI, Government Response Severity Index; #YGLs, number of Young Global Leaders

Period	March 1, 2020, to April 30, 2020		December 1, 2020, to January 31, 2021		March 1, 2020, to January 31, 2021	
Variables	Coefficient	p-value	Coefficient	p-value	Coefficient	p-value
Intercept	74.6±2.3	<2×10^-16^	46.4±2.4	<2×10^-16^	58.0±2.2	<2×10^-16^
Weighted #YGLs in business	-0.23±0.20	0.247	0.033±0.20	0.873	-0.05±0.19	0.812
Weighted #YGLs in politics	1.2±2.2	0.588	0.86±2.3	0.704	0.18±2.1	0.932
Weighted #YGLs in civic society	1.8±2.2	0.419	1.7±2.2	0.440	2.1±2.1	0.321
Continent						
Asia vs. Africa	1.8±3.4	0.609	10.8±3.5	0.0027*	2.9±3.3	0.380
Europe vs. Africa	2.1±3.4	0.550	16.4±3.5	7.3×10^-6^*	-2.7±3.3	0.409
North America vs. Africa	6.3±4.2	0.140	9.4±4.3	0.032	4.4±4.0	0.275
Oceania vs. Africa	0.13±6.6	0.984	-5.2±6.9	0.446	-12.1±6.3	0.057
South America vs. Africa	9.2±5.3	0.085	18.9±5.5	0.00069*	18.6±5.1	0.00033*
Model fit						
R^2^	0.0317		0.181		0.130	
adj. R^2^	-0.013		0.143		0.090	
p-value (F-test)	0.683		2.6×10^-5^*		0.00183*	
AICc	1547.2		1554.3		1530.2	

Because the total number of YGLs was significantly associated with the median GRSI during the second wave and first year of the pandemic (Table 2), we also fitted regression models using this variable as a predictor. Generalized variance inflation factors between total number of YGLs and continents were small (1.0296) and thus indicated negligible collinearity between these variables. We did not assume that the correlation between YGLs and stringency of NPIs would follow a linear relationship; rather, we fitted three polynomial models with up to four degrees in addition to a linear model and identified the best-fitting model as the one having the lowest AICc. The AICc values revealed that a four-degree and two-degree polynomial provided the best model fits for the timeframes between December 2020 and January 2021 and between March 2020 and January 2021, respectively (Table 6). The number of YGLs was a significant predictor of the median GRSI during December 2020 and January 2021 in the four-degree polynomial model. Figure 2 shows the dour-degree polynomial compared to the linear model for the example of Europe. As we can see in this figure, there is a dearth of data points in the region beyond 30 YGLs per country that might have influenced the behavior of the model fits. In fact, only eight of the 182 countries (4.3%) had more than 30 YGLs (China, Germany, India, Japan, Singapore, Switzerland, the United Kingdom, the USA). We therefore decided to refit linear regression models on a dataset that excluded these eight countries with more than 30 YGLs. The results for testing hypothesis H3 on this dataset as well as for the regression on the total number of YGLs are given in Table 7 and Table 8, respectively.

**Table 6:** Best-fit regression models for predicting the median GRSI in three time periods using total number of YGLs as a predictor For each period, the displayed model is the best-fit model from a set of four polynomial models of increasing degree (from linear to fourth degree). *p<0.01 (statistically significant). AICc, bias-corrected Akaike Information Criterion; GRSI, Government Response Severity Index; #YGLs, number of Young Global Leaders

Period	March 1, 2020, to April 30, 2020		December 1, 2020, to January 31, 2021		March 1, 2020, to January 31, 2021	
Variables	Coefficient	p-value	Coefficient	p-value	Coefficient	p-value
Intercept	74.9±2.3	<2×10^-16^	44.8±2.4	<2×10^-16^	57.9±2.2	<2×10^-16^
Total #YGLs	-0.03±0.05	0.574	1.49±0.51	0.0036*	0.27±0.13	0.042
(Total #YGLs)^2^	−	−	-0.047±0.021	0.026	-0.0008± 0.00046	0.085
(Total #YGLs)^3^	−	−	0.0004±0.0002	0.041	−	−
(Total #YGLs)^4^	−	−	-9.0×10^7^± 4.5×10^-7^	0.048	−	−
Continent						
Asia vs. Africa	1.7±3.4	0.607	8.2±3.5	0.022	1.3±3.3	0.685
Europe vs. Africa	2.5±3.4	0.465	14.8±3.5	3.8×10^-5^*	-3.3±3.3	0.306
North America vs. Africa	6.1±4.2	0.150	9.4±4.2	0.027	4.4±4.0	0.273
Oceania vs. Africa	0.05±6.6	0.993	-6.1±6.7	0.423	-12.8±6.3	0.043
South America vs. Africa	9.3±5.3	0.079	15.9±5.4	0.0037*	17.8±5.0	0.00049*
Model fit						
R^2^	0.0259		0.223		0.142	
adj. R^2^	-0.0075		0.183		0.108	
p-value (F-test)	0.591		1.2×10^-6^*		0.00033*	
AICc	1543.9		1551.1		1525.5	

**Figure 2:** Best-fitting model to predict the median GRSI between December 2020 and January 2021 with the total number of YGLs in a European country (blue) compared to the linear model fit (red). GRSI, Government Response Severity Index; YGLs, Young Global Leaders

**Table 7:** Regression models for predicting the median GRSI in three time periods according to hypothesis H3 on the dataset excluding countries with more than 30 YGLs *p<0.01 (statistically significant). AICc, bias-corrected Akaike Information Criterion; GRSI, Government Response Severity Index; #YGLs, number of Young Global Leaders

Period	March 1, 2020, to April 30, 2020		December 1, 2020, to January 31, 2021		March 1, 2020, to January 31, 2021	
Variables	Coefficient	p-value	Coefficient	p-value	Coefficient	p-value
Intercept	74.6±2.4	<2×10^-16^	45.6±2.4	<2×10^-16^	58.0±2.2	<2×10^-16^
Weighted #YGLs in business	0.37±0.81	0.646	2.05±0.84	0.016	1.53±0.78	0.052
Weighted #YGLs in politics	1.2±2.6	0.660	-2.7±2.7	0.317	-2.3±2.5	0.932
Weighted #YGLs in civic society	-0.66±3.8	0.864	-1.2±4.0	0.764	-0.16±3.7	0.964
Continent						
Asia vs. Africa	2.1±3.5	0.545	8.9±3.7	0.016	1.4±3.4	0.684
Europe vs. Africa	1.9±3.5	0.580	15.3±3.6	3.3×10^-5^*	-3.4±3.3	0.311
North America vs. Africa	5.7±4.2	0.172	9.8±4.3	0.025	4.6±4.0	0.249
Oceania vs. Africa	-0.4±6.6	0.951	-5.7±6.8	0.407	-12.6±6.3	0.049
South America vs. Africa	8.5±5.3	0.111	17.5±5.4	0.0017*	17.4±5.1	0.00078*
Model fit						
R^2^	0.0313		0.181		0.155	
adj. R^2^	-0.016		0.143		0.114	
p-value (F-test)	0.721		2.6×10^-5^*		0.00414*	
AICc	1475.9		1488.7		1460.8	

**Table 8:** Linear regression models for predicting the median GRSI in three time periods using total number of YGLs as a predictor on the dataset excluding countries with more than 30 YGLs AICc, bias-corrected Akaike Information Criterion; GRSI, Government Response Severity Index; #YGLs, number of Young Global Leaders *p<0.01 (statistically significant).

Period	March 1, 2020, to April 30, 2020		December 1, 2020, to January 31, 2021		March 1, 2020, to January 31, 2021	
Variables	Coefficient	p-value	Coefficient	p-value	Coefficient	p-value
Intercept	74.9±2.3	<2×10^-16^	45.5±2.4	<2×10^-16^	57.4±2.2	<2×10^-16^
Total #YGLs	-0.03±0.05	0.574	0.66±0.24	0.0063*	0.51±0.22	0.021
Continent						
Asia vs. Africa	1.7±3.4	0.607	9.0±3.6	0.013	1.3±3.3	0.699
Europe vs. Africa	2.5±3.4	0.465	15.3±3.6	2.9×10^-5^*	-3.5±3.3	0.291
North America vs. Africa	6.1±4.2	0.150	9.3±4.3	0.032	4.1±4.0	0.297
Oceania vs. Africa	0.05±6.6	0.993	-6.3±6.8	0.353	-13.2±6.3	0.036
South America vs. Africa	9.3±5.3	0.079	17.3±5.4	0.0018*	17.0±5.0	0.00085*
Model fit						
R^2^	0.0259		0.194		0.153	
adj. R^2^	-0.0075		0.165		0.122	
p-value (F-test)	0.591		2.2×10^-6^*		9.4×10^-5^*	
AICc	1543.9		1484.8		1456.9	

## Discussion

Summary

We found in this correlational study that the absolute number of YGLs trained by the WEF since 2016 correlated significantly with a Spearman’s ρ > 0.30 with a country’s median and maximum strength of the implemented NPIs during the second wave of the Covid-19 pandemic, but not during the first wave. This correlation was larger than the prespecified threshold of ρ = 0.30 and clearly significant with p < 2×10^-6^ (Table 2 and Table 3). This association was non-linear with a fourth-degree polynomial model representing this non-linear relationship best, together with differential effects over continents (Table 6). This model is highly significant (p <2×10^-6^), and explains roughly 18% of the variance. Our differential hypothesis, namely that more influential leaders or different types of leaders would have a different effect was not supported (Table 5 and Table 7).

Interpretation

Correlation is not causation, yet correlations are preconditions for causation. Our data might therefore be interpreted along the following lines: The WEF is a large amplifier network, as it has trained YGLs across the world, that is, in most countries and especially in those considered to be among the most economically important ones. Out of the 182 countries with data on NPIs, 102 hosted at least one global leader; thus roughly 60% of all countries in the world are home to at least one YGL, and eight countries hosted more than 30 YGLs. If the WEF has formed a coherent opinion on the crisis as well as on the corresponding mitigation measures, then this opinion may have been shared and amplified by the YGL network. In fact, our data suggest that this has been the case after the first wave. Thus, the network might have operated as a selector and an echo chamber for shared, politically desirable opinions which were then amplified and propagated through the network.

Notably, however, there is no association between the number of YGLs per country and the strength of the NPIs during the first wave of the pandemic. This suggests that the WEF did not play a role in determining the scale and scope of the NPIs implemented in the initial stages of the pandemic. Thus, it seems as if this phase has been driven by other factors, such as recommendations by the WHO and mimicry between countries [31]. But as NPIs became established as potential pandemic mitigation measures, the WEF seems to have become a selective and reinforcing factor. In fact, the WEF has featured and advocated specific NPIs − including early prototypes of the later digital COVID certificates then dubbed “COVID-19 health passports”, mass scale health propaganda via ringtones, and electronic bracelets for infected or quarantined persons − as viable mitigation measures [15], and in this sense the YGLs seem to have been supportive as well [18]. Interestingly, the Young Global Business Leaders seem to have played a somewhat different role, although the observed effect is relatively weak. Still, the regression weights of the YGLs in business were small and negative during the first wave as well as throughout the entire period (Table 5), whereas those in politics and civil society had a large and positive regression weight. This supports the idea that the WEF does not have a uniform message.

One might argue that the non-linearity is an artifact of a few outlier countries. We tested this by a restricted linear model excluding outlier countries (Table 8) and found a linear relationship which was also significant, the model explaining roughly 17% of the variance. In addition, continents played also a role: NPIs were more strongly implemented in Europe and South America.

Reverse causality is an unlikely explanation: YGLs were trained before the pandemic, and the pandemic did not have an influence on the distribution of YGLs across countries, not least because the selection process of YGLs is entirely managed by the WEF administration itself [16,17].

There could, of course, be numerous other variables not taken into consideration in this study that might be drivers of the correlation between number of YGLs and NPIs in a country. For instance, countries with more YGLs might also be in closer diplomatic contact and hence have similar outlooks on issues related to the implementation of NPIs. But it seems unlikely that such diverse countries as Afghanistan (five YGLs), Sweden (three YGLs), Sri Lanka (three YGLs), and Ukraine (three YGLs) would coordinate their NPIs through direct diplomatic contacts. It is rather conceivable that YGLs do exert the influence anticipated by the WEF while training and after having trained them: by informally, perhaps also formally, influencing the policies and public opinion in their countries.

A vignette might support this: Uruguay (one YGL) and Argentina (11 YGLs) are neighboring countries with a similar population density (Argentina 16 inhabitants per km2, Uruguay 20 per km2), although their total population size is very different. While Argentina imposed one of the most severe lockdowns, Uruguay did not, and fared much better for whatever reasons [32].

Our data refute the idea that the WEF had been planning or otherwise stage-managing the crisis, as the correlation between YGLs and NPIs was non-existent during the first wave of the pandemic. This is despite the fact that the WEF took part in major pandemic preparedness exercises such as Event 201 [19] and holds relations with other NGOs and pharmaceutical companies that have been implicated in “planning” the COVID-19 crisis [28]. The strength of the correlation grew during the first year of the pandemic to a sizeable and significant strength of around ρ = 0.30 from October 2020 onward. Since we were only interested in the first phases of the pandemic, we did not test for further developments, although these might be interesting. Initially, other processes seem to have driven the implementation and severity of NPIs. It is likely that the YGL community is in mutual exchange and hence coordinates and mainstreams opinions and political outlooks. It is interesting to observe that after the first wave, some studies were published that were factually wrong, suggesting that lockdowns were useful, for instance Dehning et al. [33] in the case of Germany who were later shown to be wrong [3]. Critical voices warning of the sensitivity of initial parameters in supportive models went often unheard [34]. This seems to have happened because a mainstream opinion had already been established across many countries that also defined what was considered politically correct and good for everyone’s health. This is the typical domain of shaping public opinion despite a lack of, or even in the face of, contradicting evidence. And this might be indeed associated with YGL influence in a country as one influential factor among many others. A study like ours is only able to scratch at the surface on the question of unwarranted interference of the WEF and its global network in the affairs of civil society and public health in what appears to be a controlled demolition of democratic rights [4,9]. Since the WEF exists since 1971 [12], subsequent studies might attempt to longitudinally analyze how the WEF has managed through the decades to gain such control over governments, corporations, and the media.

Our data are deliberately coarse-grained, as we thought that only a really robust effect is worthwhile considering. One might have improved the resolution by defining individual waves per country and by adapting the correlations accordingly as in Hale et al. [8]. We would assume that such a finer resolution would rather strengthen than weaken our findings.

We considered some, but clearly not all potential additional factors, such as population size and continent. They did not alter the picture substantially. It would be interesting to add other variables such as mortality rates, preparedness of medical systems, number of intensive care unit beds per 1,000 inhabitants, and similar variables to see whether our correlation between YGLs and NPIs in a country is explainable by other factors.

Our results are not due to an exploratory fishing expedition: We defined our procedures and the analyses in advance, as much as possible in an open project like this. For instance, we did not explore different time windows and report only on those where we found significant results. We calculated the three reported correlations and explored them in a modeling approach. We defined what we call “significant correlation” in our protocol before we started the analysis. Hence, our results are robust and not likely to be a chance correlation. In fact, that likelihood is given by our significance level and is smaller than 2×10^-6^. This is more than 5 sigma, an effect level that is rare in medical and social contexts, and would be called an “effect” within the physics community [35]. Our analysis explains 18% of the variance. This is sizeable, but leaves room for many other factors to be considered.

Limitations

We only considered the YGL data of the last five years because we assumed that YGLs trained further in the past might not be as relevant as the ones from the more recent past. This might not be the case. This is a secondary study, and our results are only as good as the original data. In order to prove causality, we would have to study mechanisms in depth. This is obviously very complicated and would only be possible by further anthropological and qualitative approaches, which are beyond our resources. One possibility would be to utilize Critical Discourse Analysis [36] to study the public discourse key rhetorical devices for hints towards collusion among YGLs.

## Conclusions

Restating our research question “*Is the number and the gravitas of YGLs in a country associated with the country’s NPI in the first phases of the pandemic in 2020?*” we conclude that there was an association between the number of YGLs in a country and a country’s strength of NPIs during the second phase of the pandemic, but not during the first. This speaks in favor of the hypothesis that the WEF operates as an amplifier network or an echo-chamber for certain opinions that might either be presented to the network or that might arise within it and be then transported through it. More qualitative studies should be undertaken to identify putative causal mechanisms underlying our observed correlations.
